# Comparison of the Effects of Open Surgery and Minimally Invasive Surgery on the Achilles Tendon Rupture Healing Based on Angiogenesis

This article has been retracted.

**DOI:** 10.1155/2022/1447129

**Published:** 2022-09-01

**Authors:** Fan Gong, Xiaoliang Li, Hanling Zhang, Jianke Wu, Guoxu Ma, Bowen Zhang, Jian Gao, Yi Ding, Yonglu Huang, Suoli Cheng, Xuebing Zhou, Fei Zhao

**Affiliations:** Hand & Foot & Reconstruction Microsurgery, People's Hospital of Ningxia Hui Autonomous Region (The First Affiliated Hospital of Northwest University for Nationalities), Yinchuan 750002, Ningxia, China

## Abstract

**Objective:**

To compare the effect of three different surgical methods on rabbit Achilles tendon rupture.

**Methods:**

The Achilles tendon transection model was constructed by cutting off the inner half of the Achilles tendon. Rabbits were divided into 4 groups: model group, open surgery (OS) group, minimally invasive surgery (MS) group, and conservative treatment (CT) group. Biomechanical evaluation, H&E, and Picrosirius Red staining were applied to evaluate the histological changes and healing. RT-qPCR, Western blot, ELISA, and IHC staining were used to detect the expression of COLIII, IL-1*β*, TNF-*α*, IL-6, CD31, VEGF, bFGF, and TGF-*β*1.

**Results:**

Different surgery treatments significantly alleviated the histological changes in rabbits. The tension and elasticity of the Achilles tendon were significantly increased after surgery. In addition, surgery treatments notably alleviated the inflammatory responses *in vivo* via downregulation of IL-1*β*, TNF-*α*, and IL-6 and promoted the tube formation in tissues through upregulating VEGF, bFGF, TGF-*β*1, and CD31. Furthermore, MS exhibited best therapeutic efficiency on Achilles tendon rupture healing, compared with OS or CT.

**Conclusions:**

Our research revealed the superiority of MS in Achilles tendon rupture treatment at the molecular level compared with OS or CT.

## 1. Introduction

Achilles tendon rupture is a subtype of the prevalent tendon injuries [1, 2]. Most of the injuries happen in sports exercise, and the prevalence of injuries has been increasing among the sports participants [3, 4]. Nowadays, excessive strenuous exercise and repeated local inflammation can lead to the rupture of the Achilles tendon [5]. The clinical treatment outcome of Achilles tendon rupture is ideal due to the adopted surgical or nonsurgical treatments. However, the return to the sports before sufficient maturation of tendon can lead to repeat rupture, and this happens in 4.5%–12% and 2.8%–7.1% of cases after conservative treatment and surgeries, respectively [6].

Tendon healing includes overlapping and mutually dependent proliferative, inflammatory, and remodeling stages. Inflammatory cells and erythrocytes enter the injury site during the initial inflammatory phase. Meanwhile, macrophages and monocytes often phagocytose the necrotic tissues in this phase. Then, the release of growth factors can promote the proliferation and angiogenesis of fibroblasts, and this phenomenon can lead to the migration of fibroblasts to the injury site. After that, the synthesis of type III collagen is initiated. The synthesis of type III collagen usually remains increased for about 42 days during the proliferative phase. Moreover, a bigger proportion of type I collagen is synthesized in the subsequent remodeling phase [7, 8].

At present, there are three major types of Achilles tendon rupture repair surgery: open surgery (OS), minimally invasive surgery (MS), and conservative treatment (CT). Each of these surgical methods has advantages and disadvantages. For example, a previous study reported that the quality of healing after conservative treatment is poor, and the possibility of breaking again is also high [9]. Meanwhile, the side effect of CT is known to be limited, while the recovery period is too long [10]; the recovery period of MS is relatively short, and the side effect of MS is less obvious compared with OS [4, 11]. According to these studies, MS appears to be more conducive to the rupture and healing of the Achilles tendon, with less surgical injury and faster postoperative recovery. However, which surgical method is more efficient is not clear.

Thus, our study aimed to explore the efficiency of these three surgeries based on angiogenesis, as well as to investigate the underlying mechanism at molecular level. We hope our work would shed new light on finding the ideal treatments for rupture of the Achilles tendon.

## 2. Materials and Methods

### 2.1. Animal Model

The rabbit model of Achilles tendon rupture was constructed as recently described [12]. Thirty-two New Zealand white rabbits (SPF, half male half female, three-month-old, 3.5 ± 0.4 kg, Guangdong Medical Laboratory Animal Center, China) were raised in a pathogen-free environment, alternating light and dark for 12 h (8:00 am–8:00 pm). This experiment was carried out in accordance with the animal experiment guidelines, and the research plan was approved by the Animal Experiment Committee.

Rabbits were divided into four groups: model, MS, OS, and CT (*N* = 8, half male half female). All rabbits were modeled with Achilles tendon rupture. Model groups were not processed after modeling. The remaining groups were treated according to the group method.

Sodium pentobarbital (20 mg/kg body weight) was used to inject intravenously into the rabbits, and then we shaved the skin of right hind limb. The procedure of surgeries was used under the aseptic condition. The midline of the Achilles tendon was cut longitudinally with a gap. Subsequently, the paratenon was cut, and we then dissected the tendon of Achilles and plantaris from the surrounding tissues. After that, a scalpel was applied to cut off the middle of the Achilles tendon. The plantaris tendon was left intact as an internal splint. The severed tendon was not sutured. All models were performed on the right hind legs, and the left hind legs were used as an internal reference.

The rabbits in the CT group were treated with plaster to avoid movement. Rabbits in the OS group were treated with open sutures. After disinfection, the Achilles tendon was sutured directly by incising the skin, and then the skin was sutured layer by layer. In the MS group, minimally invasive suture was performed percutaneously. In brief, the ruptured Achilles tendon was sutured minimally through two proximal and two distal puncture routes. Suture line was Vicryl® (3.0, Polyglactin 910, Ethicon, USA). The recovery of the Achilles tendon in the early stage of healing (6 w) was analyzed.

### 2.2. Biomechanical Evaluation

Both ends of the left and right Achilles tendons of each rabbit were fixed on a test device (Lloyd, LS500, England). After fixing, a tensile test (10 mm/min) was performed. 1 kN electromechanical sensor (MTS Synergie, Eden Prairie, MN, USA) was applied to detect the stress-strain curve, and the elastic modulus (MPa) and failure stress (MPa) were calculated. The maximum force (N) required to break each sample was recorded as load until failure. For each rabbit, the percentage of the experimental side (right side, named treatment) to the health test (left side, named not treated, NT) was calculated.

### 2.3. H&E and Picrosirius Red Staining

The Achilles tendon tissue at the edge of the healing site was used for histological evaluation. The tissues were fixed (neutral formalin, 10%), sectioned, and deparaffinized. Hematoxylin was added and incubated at room temperature for 10 min, then 0.5% eosin solution was added and incubated at room temperature for 3 min. For the evaluation of collagen formation, Picrosirius Red solution was used to stain for 1 h. After washing and dehydrating, neutral gum was used to seal. The samples were observed under microscope (Olympus, Japan) at × 100 magnification.

### 2.4. ELISA

IL-6 ELISA kit (PI335, Beyotime, China) and IL-1*β* (ml02783) and TNF-*α* ELISA kit (ml001696, Mlbio, China) were used to detect. Achilles tendon tissues at the edge of the healing site were triturated and lysed, and the supernatant was collected by centrifugation (1,000 x g, 4°C). Into each 96-well plate, 100 *μ*l of sample was added. Then, 100 *μ*l enzyme-labeled reagent was added and incubated at 37°C for 1 h. Subsequently, 50 *μ*l of chromogenic reagent A was added into each well and an equal volume of chromogenic reagent B was added. The mixture was shaken gently to mix the two stains evenly in the dark. After 15 min, 50 *μ*l stop solution was added to the reaction to halt color development. It was observed that the sample color changed from blue to yellow. Subsequently, the absorbance was detected. A blank well was used for zero adjustment and the detection wavelength used was 450 nm (680, Bio-Rad, USA). A standard curve was used to determine the concentrations of IL-6, IL-1*β*, and TNF-*α*.

### 2.5. Reverse Transcription-Quantitative PCR (RT-qPCR)

In the early stage of healing (6 weeks postoperatively), the Achilles tendon tissues at the edge of the healing site were collected, and TRIzol® reagent (Thermo Fisher Scientific) was applied to extract total RNA from tissues. Then, total RNA was reverse transcribed into complementary DNA (cDNA), followed by RT-qPCR examination using SYBR Green Master Mix on the ABI 7900 Real-Time PCR System. Real-time qPCRs were performed in triplicate under the following protocol: 94°C for 2 minutes, followed by 35 cycles (94°C for 30 s and 55°C for 45 s). The primer pairs were as follows: COLIII forward, 5′-TCACTGGTCTTTTGGAGTTT-3′ and reverse, 5′-GTGAGGAACAAGCCAGAGCT-3'; IL-6 forward, 5′-AAACTCTGCAAGATGCCACA -3′ and reverse, 5′-GTCTGAGGCTCATTCTGCCC -3'; IL-1*β* forward, 5′-GCAGGCACAGAACCAGTGGC-3′ and reverse, 5′-GGAGTTCCTGCAGTCCAGCC -3'; TNF-*α* forward, 5′-ATGTTGTTCTCTATGGAGAA-3′ and reverse, 5′-AATTTATTAATATTTAAATA -3'; VEGF forward, 5′-CCTCAAATAAATGGCTAACT-3′ and reverse, 5′-AATGTATAAATGGTTTTTAT-3'; bFGF forward, 5′-TCTTGGAAAGTGTAGGCTTA-3′ and reverse, 5′-TATTTATATTGTATTTATAT-3'; *β*-actin forward, 5′-GTCCACCGCAAATGCTTCTA-3′ and reverse, 5′-TGCTGTCACCTTCACCGTTC-3'. The 2^−ΔΔct^ method was used to quantify the data. *β*-Actin was applied for normalization.

### 2.6. Western Blotting

The Achilles tendon tissue at the edge of the healing site was lysed using RIPA lysis buffer (Beyotime). Equal amounts (20 *μ*g) of protein from each group were separated by SDS-PAGE electrophoresis. Separated proteins were transferred on to a PVDF membrane. Then, primary antibodies against COLI (ab239007, 1:1000, Cambridge, MA, USA), COLIII (ab239007, 1:1000), and GAPDH (ab179467, 1:1000) after blocking and HRP-conjugated secondary antibodies (Abcam; ab7356, 1:5000) were used to incubate with the membrane. All the antibodies were obtained from Abcam (MA, USA). ECL kit (Thermo Fisher Scientific) was applied to visualize the protein bands. *β*-Actin was used for normalization. The densitometry analysis was performed by IPP 6.0 (Image-Pro Plus 6.0).

### 2.7. Immunohistochemical (IHC) Staining

The Achilles tendon tissue at the edge of the healing site of rabbits was fixed, paraffin-embedded, and cut into sections (5 *μ*m thick). Paraffin sections were deparaffinized and rehydrated. Subsequently, the sections were heated, incubated for 25 min in 3% H_2_O_2_, washed, blocked, and incubated for 30 min. After that, primary antibodies (anti-CD31 and anti-VEGF) were applied to stain the samples overnight. Samples were treated with HRP-labeled secondary antibody. After 30 min of incubation, diaminobenzidine (DAB) was applied for the development of color. All the antibodies originated from Abcam.

### 2.8. Statistical Analysis

Three independent experiments were performed in each group, and the mean ± standard deviation (SD) was used to express all data. Difference between the two groups was analyzed using Student's t-test. Differences between the groups were performed using one-way analysis of variance (ANOVA) and Tukey's test (Graphpad Prism7). A significant difference was indicated by the result of *P* < 0.05.

## 3. Results

### 3.1. MS Alleviates the Injury and Promotes the Recovery Biomechanical Indicators of the Achilles Tendon Rupture Tissues

To compare the efficiency of three different surgeries for Achilles tendon rupture, H&E staining was performed. It was showed after 1 and 6 weeks of surgery, fibroblasts and angiogenesis in tissues of rabbits were significantly increased, while inflammatory infiltration (including inflammatory cells) was obviously alleviated. Meanwhile, the phenomenon after 6 weeks was more obvious, compared with 1 week. Furthermore, MS exhibited better anti-inflammatory and pro-angiogenesis effect to the ruptured Achilles tendon tissues, compared with OS and CT treatment (Figure 1). Thus, the above results demonstrated that MS treatments could effectively alleviate the injury of the Achilles tendon rupture tissues in a rabbit model.

In addition, 6 weeks after modeling, the elastic modulus, failure stress, and load until failure indicators after OS and MS treatment all increased significantly (Figures 2(a)–2(c)). Moreover, the biomechanical indexes of the MS group were significantly higher than those of the OS group (Figures 2(a)–2(c)). This suggested that both OS and MS treatment could effectively restore the elasticity and strength of the Achilles tendon in the early stage, and the effect of MS was more significant.

### 3.2. MS Attenuates the Inflammatory Responses of the Achilles Tendon Rupture Tissues in a Rabbit Model

Next, we investigated the effect of different surgeries on inflammatory responses in Achilles tendon tissues. The data showed that the mRNA of IL-1*β*, TNF-*α*, and IL-6 in tissues of rabbits was significantly downregulated in the model group (Figures 3(a)–3(c)). All three surgical methods could effectively reduce the level of these inflammatory cytokines, and MS exerted the better anti-inflammatory effect compared with CT and OS. Similarly, the data of ELISA demonstrated that three surgical methods significantly decreased the level of IL-1*β*, TNF-*α*, and IL-6 in tissues of rabbits, and MS exhibited the most anti-inflammatory effect (Figures 3(d)–3(f)). Taken together, all these data revealed that MS significantly attenuated the inflammatory responses in Achilles tendon rupture tissues of rabbits.

### 3.3. MS Significantly Promotes the Angiogenesis of the Achilles Tendon Rupture Tissues in a Rabbit Model

In order to further analyze the molecular mechanisms affecting the healing of Achilles tendon rupture, this study firstly detected the levels of growth factors TGF-*β*1 and bFGF. The results showed that the levels of TGF-*β*1 and bFGF mRNA in tissues of rabbit model were greatly upregulated in three treatment groups compared with the model group (Figures 4(a) and 4(b)), while the CT group exhibited the lowest expression of TGF-*β*1 and bFGF mRNA compared with OS and CT groups. Moreover, the levels of TGF-*β*1 and bFGF mRNA in the MS group were significantly higher than those in the OS group (Figures 4(a) and 4(b)). These growth factors not only promoted the proliferation and differentiation of tissue cells but also participated in the induction of angiogenesis and promoted blood perfusion at the injured site. In this study, CD31 and VEGF were used to assess the growth of blood vessels. The results of IHC experiments showed that the CD31 and VEGF proteins in CT, OS, and MS groups all increased to varying degrees. The CD31 and VEGF levels of OS and MS group were significantly higher than those of the CT group. The MS group had the highest expression of CD31 and VEGF proteins (Figures 4(c)–4(e)). This suggested that compared to OS, MS was more helpful in retaining growth factors and promoting angiogenesis in the early stages of healing.

### 3.4. MS Significantly Promotes the Healing of the Achilles Tendon Rupture Tissues in a Rabbit Model

In the early stage of Achilles tendon repair, fibroblasts gradually migrated to the injury site and expressed COLIII. The up-regulation of the COLIII expression level within 6 weeks could reflect the early repair of Achilles tendon. The level of COLIII at 6 weeks could reflect the early repair of the Achilles tendon. The results indicated that three different treatments significantly upregulated the expressions of COLIII in Achilles tendon tissues at both mRNA and protein levels (Figures 5(a) and 5(b)). Furthermore, the effects of MS on COLIII mRNA and protein expressions were more significant, compared with CT and OS (Figures 5(a) and 5(b)). In addition, the results of Picrosirius Red staining showed that after treatment, the degree of fibrosis in the three groups was significantly increased. Among them, the fibers of the MS group were the most uniform and abundant (Figure 5(c)). This showed that at 6 weeks after surgery, MS was most conducive to the repair of Achilles tendon fibrosis.

## 4. Discussion

The main function of the Achilles tendon is flexion of the calf and foot extension. Once the Achilles tendon ruptures, it will seriously affect the patient's exercise ability and cause great inconvenience to the patient's daily life. There are two main treatments for closed Achilles tendon rupture: nonsurgical treatment (conservative treatment) and surgical treatment [13, 14]. The biggest complication of nonsurgical treatment is that the Achilles tendon is more likely to be broken again. At the same time, it requires a long time for plaster immobilization, which seriously affects the patient's quality of life [15, 16]. The surgical treatment is generally divided into two types: OS and minimally invasive surgery. OS has always been the “gold standard” for Achilles tendon rupture. However, scarring is easy to form after OS, and complications such as necrosis of the surrounding skin and exposure to Achilles tendon may occur [17–19]. The purpose of percutaneous surgery is to reduce the rate of re-fracture of the heel key and to minimize infection and soft tissue complications [20, 21]. MS also has some disadvantages. The broken form of the heel key is complicated and irregular, so percutaneous or minimally invasive surgery cannot be well exposed and repaired.

However, there are no systematic reports and studies in the literature that these two surgical methods are more effective. In addition, the underlying mechanism remains unclear. The results of a latest meta-analysis show that OS is more damaging to wounds, while MS seems to be more helpful in the early repair of Achilles tendon, and the long-term efficacy of the two is not significantly different [22]. In order to evaluate the effects of OS and MS on the early healing of Achilles tendon rupture, rabbits were used for experimental analysis. The results show that 6 weeks after modeling, both OS and MS can promote the healing of the ruptured Achilles tendon, and MS more effectively restores the elasticity and bearing capacity of the Achilles tendon. In addition, the results also show that MS treatment can effectively inhibit the levels of inflammatory cytokines and promote the expression of growth factors TGF-*β*1 and bFGF. Moreover, the results of this experiment also show that the repaired tissues of CT, MS, and OS groups all have the expression of VEGF and CD31 protein, while the levels of VEGF and CD31 in the MS group are the highest, suggesting that the blood vessels are the most abundant. Surgery can cause local ischemia and stress damage and promote the increase of inflammatory cytokines, which cause the loss of growth factors and inhibit angiogenesis [18]. This suggests that MS may accelerate Achilles tendon repair by promoting angiogenesis in the early stage of repair.

VEGF (approximately 45 kDa) is a homodimeric glycoprotein [23]. It plays a vital role in angiogenesis. In addition, it can bind VEGF receptor-1 and VEGF receptor-2, which are distributed in vascular endothelial cells [24]. Meanwhile, VEGF can induce angiogenesis in the development of embryo, which is crucial in wound healing in healthy adults [25]. In this research, we found that the surgery treatment could promote the angiogenesis, and it could upregulate the expression of VEGF. Previous studies indicated that VEGF upregulation could promote angiogenesis [26, 27]. VEGF and COLIII have a synergistic effect, and they work together to promote wound repair [28]. COLIII is a key protein for early Achilles tendon fibrosis, and it continues to increase within 6 weeks after healing [29–31]. The increase of COLIII indicates that the early healing degree is good and the speed is fast. The results of this study show that, corresponding to angiogenesis, the MS group also has the highest COLIII level. The function maintenance and repair of tendons are inseparable from the joint action of VEGF and COLIII [32]. In vitro study shows that VEGF can promote the expression of COLIII and promote fibrosis [33]. Based on this, the results of this study show that MS may promote the early repair of Achilles tendon rupture by promoting angiogenesis and the expression of COLIII, thereby accelerating healing. The expression of VEGF, COLIII, and other genes by different treatments may be related to the different effects of trauma, tissue repair, and subsequent inflammation. The mechanisms by which different treatments affect gene expression require in-depth studies.

MS has the advantages of both OS and CT. Compared with CT, MS can effectively repair the Achilles tendon and avoid the postoperative scarring and inflammation problems associated with OS.

## 5. Conclusion

In conclusion, MS, OS, and CT significantly promoted the repair of Achilles tendon injury. In addition, the anti-inflammatory and pro-angiogenesis effect of MS was much better than other two treatments; the levels of COLIII (fibrotic markers) were more sensitive to MS, compared with CT and OS, suggesting that MS exhibited more significant therapeutic effects on Achilles tendon rupture, compared with CT and OS. Therefore, our study might shed new light on exploring the best methods for Achilles tendon rupture surgery. However, there is a big difference between animal research and human research. The mechanism by which MS promotes angiogenesis still needs to be studied in depth.

## Figures and Tables

**Figure 1:** CT, OS, and MS alleviate the injury of the Achilles tendon rupture tissues. After 1 or 6 weeks of surgeries, the histological changes in Achilles tendon tissues of rabbits were observed by H&E staining.

**Figure 2:** CT, OS, and MS promote the recovery biomechanical indicators of the Achilles tendon rupture tissues. (a) The effect of CT, OS, and MS on the elastic modulus of Achilles tendon. (b) The effect of CT, OS, and MS on the failure stress of Achilles tendon. (c) The effect of CT, OS, and MS on the failure stress of Achilles tendon. _ _^*∗*^*P* < 0.05, *P*^*∗∗*^ < 0.01, and  ^*∗∗∗*^*P* < 0.001 compared to model. _ _^#^*P* < 0.05, _ _^##^*P* < 0.01, and _ _^###^*P* < 0.001 compared to CT. _ _^∧^*P* < 0.05,  ^∧∧^*P* < 0.01, and  ^∧∧∧^*P* < 0.01 compared to OS.

**Figure 3:** MS attenuates the inflammatory responses of the Achilles tendon rupture tissues in a rabbit model. The expressions of (a) IL-6, (b) TNF-*α*, and (c) IL-1*β* in Achilles tendon tissues of rabbits were detected by RT-qPCR. The levels of (d) IL-6, (e) TNF-*α*, and (f) IL-1*β* in Achilles tendon tissues of rabbits were detected by ELISA. _ _^*∗*^*P* < 0.05,  ^*∗∗*^*P* < 0.01, and  ^*∗∗∗*^*P* < 0.01 compared to model. _ _^#^*P* < 0.05, _ _^##^*P* < 0.01, and _ _^###^*P* < 0.001 compared to CT. _ _^∧^*P* < 0.05,  ^∧∧^*P* < 0.01, and  ^∧∧∧^*P* < 0.01 compared to OS.

**Figure 4:** MS significantly promotes the angiogenesis of the Achilles tendon rupture tissues in a rabbit model. (a, b) The levels of bFGF and TGF-*β*1 mRNA in Achilles tendon tissues of rabbits were detected by RT-qPCR. (c, d, e) The protein levels of CD31 and VEGF in Achilles tendon tissues of rabbits were tested by IHC staining. _ _^*∗*^*P* < 0.05, *P*^*∗∗*^ < 0.01, and  ^*∗∗∗*^*P* < 0.01 compared to model. _ _^#^*P* < 0.05, _ _^##^*P* < 0.01, and _ _^###^*P* < 0.001 compared to CT. _ _^∧^*P* < 0.05,  ^∧∧^*P* < 0.01, and  ^∧∧∧^*P* < 0.01 compared to OS.

**Figure 5:** MS significantly promotes the healing of the Achilles tendon rupture tissues in a rabbit model. (a, b) The expressions of COLIII mRNA and protein in Achilles tendon tissue of rabbits were tested by RT-qPCR and Western blot. (c) The symptom of Achilles tendon rupture was observed by Picrosirius Red staining. _ _^*∗*^*P* < 0.05,  ^*∗∗*^*P* < 0.01, and  ^*∗∗∗*^*P* < 0.01 compared to model. _ _^#^*P* < 0.05, _ _^##^*P* < 0.01, and _ _^###^*P* < 0.001 compared to CT. _ _^∧^*P* < 0.05,  ^∧∧^*P* < 0.01, and  ^∧∧∧^*P* < 0.01 compared to OS.

## Data Availability

The datasets used and analyzed during the current study are available from the corresponding author upon reasonable request.
